# Progress of Bulbar Conjunctival Microcirculation Alterations in the Diagnosis of Ocular Diseases

**DOI:** 10.1155/2022/4046809

**Published:** 2022-08-28

**Authors:** Zhengze Sun, Yaxin Li, Rongjun Liu, Baikai Ma, Yifan Zhou, Hongyu Duan, Linbo Bian, Wenlong Li, Hong Qi

**Affiliations:** ^1^Department of Ophthalmology, Peking University Third Hospital, Beijing Key Laboratory of Restoration of Damaged Ocular Nerve, Beijing 100191, China; ^2^The First Hospital of Fangshan District, Beijing 102400, China

## Abstract

Bulbar conjunctival microcirculation is a microvascular system distributed in the translucent bulbar conjunctiva near the corneal limbus. Multiple ocular diseases lead to bulbar conjunctival microcirculation alterations, which means that bulbar conjunctival microcirculation alterations would be potential screening and diagnostic indicators for these ocular diseases. In recent years, with the emergence and application of a variety of noninvasive observation devices for bulbar conjunctiva microcirculation and new image processing technologies, studies that explored the potential of bulbar conjunctival microcirculation alterations in the diagnosis of ocular diseases have been emerging. However, the potential of bulbar conjunctival microcirculation alterations as indicators for ocular diseases has not been exploited to full advantage. The observation devices, image processing methods, and algorithms are not unified. And large-scale research is needed to concrete bulbar conjunctival microcirculation alterations as indicators for ocular diseases. In this paper, we provide an update on the progress of bulbar conjunctival microcirculation alterations in the diagnosis of ocular diseases in recent five years (from January 2017 to March 2022). Relevant ocular diseases include contact lens wearing, dry eye, conjunctival malignant melanoma, conjunctival nevus, and diabetic retinopathy.

## 1. Introduction

The bulbar conjunctiva is a microvascular-rich translucent membrane that covers the sclera. Microcirculation refers to the microvessels between arterioles and venules, which is the basic functional unit of blood circulation. The bulbar conjunctival microcirculation is an uneven reticulated system adjacent to the corneal limbus, supplied primarily by the anterior ciliary artery and the palpebral artery arch. The anterior ciliary artery separates a small upper branch of the sclera 3 to 5 mm outside the corneal limbus to form a blood vessel network and is distributed in the bulbar conjunctiva. The palpebral artery arch crosses the tarsal plate and is distributed in the palpebral conjunctiva, conjunctival fornix, and bulbar conjunctiva 4 mm or more from the corneal limbus. The bulbar conjunctival microcirculation is rich in branches and anastomosis, the ratio of arterioles to venules is about 1 : 2, the diameter of microvessels is between 5 and 70 *μ*m, and the blood flow velocity is between 0.52 and 3.26 mm/s [1, 2]. A variety of ocular diseases affect the bulbar conjunctival microcirculation, and due to the translucent nature of the bulbar conjunctiva, noninvasive observations of the bulbar conjunctival microcirculation can be made.

The observation of the bulbar conjunctival microcirculation initially adopted the invasive method represented by fluorescein angiography and indocyanine green contrast and could only be made qualitatively or semiquantitatively. In 2004, minimally invasive confocal fluorescence microscopy was applied to microcirculation in vivo observations at the bulbar conjunctiva of mice [3]. Since then, noninvasive methods such as digital slit-lamps, computer-assisted intravital microscopy (CAIM), retinal function imager (RFI), orthogonal polarization spectroscopy (OPS), EyeFlow™, functional slit-lamp microscopy (FSLB), and optical coherence tomography angiography (OCTA) have emerged and enabled accurate quantitative observations combined with image processing techniques [4].

With the emergence and application of advanced bulbar conjunctival microcirculation observation equipment and new image processing techniques, bulbar conjunctival microcirculation observation has been objective, quantitative, noninvasive, and easy to operate. However, at the same time, due to the lack of unified standards between different devices and the inconsistent observation processes between laboratories, the data obtained by different laboratories are less comparable. In addition, because of the location and physiological characteristics of the bulbar conjunctiva, the bulbar conjunctival microcirculation is susceptible to multiple internal and external environmental factors, making bulbar conjunctival microcirculation alterations lack specificity.

To provide an update on the progress of bulbar conjunctival microcirculation alterations in the diagnosis of ocular diseases in recent five years, a computerized search from January 2017 to March 2022 of the online electronic database PubMed was performed, using the MeSH terms “bulbar conjunctiva” and “vessel”. More generalized complementary research regarding bulbar conjunctival microcirculation alterations was also obtained from the PubMed database. A total of 37 records were initially identified. After exclusion of nonrelevant, non-English, and duplicate studies, a total of 17 records were found eligible, all of which were included in this review. Relevant ocular diseases include contact lens wearing, dry eye, conjunctival malignant melanoma, conjunctival nevus, and diabetic retinopathy as reviewed below.

## 2. Bulbar Conjunctival Microcirculation Parameters

Commonly used bulbar conjunctival microcirculation parameters include bulbar conjunctival blood flow velocity, bulbar conjunctival vessel diameter, bulbar conjunctival blood flow rate, and bulbar conjunctival vessel density.

Bulbar conjunctival blood flow velocity is often calculated by the distance of red blood cells in several consecutive shots of the bulbar conjunctiva, and the accuracy of the measurement is interfered with by eye movements. Jo et al. [5] developed a motion correction algorithm based on deep learning, which opened up a new idea for solving the problem of motion illusion in the measurement of bulbar conjunctival blood flow velocity.

There are many ways to measure bulbar conjunctival vessel diameter, and in the early days, one or more places were manually selected on the image of the bulbar conjunctival vessels for measurement. Uji et al. [6] defined the vessel diameter index as the total area of the region representing the blood vessels in the binary image divided by the total length of the blood vessels in the vascular skeleton image. Jiang et al. [2] calculated bulbar conjunctival vessel diameter by the distance between two points at half of the maximum brightness in the vertical direction of vessels in the bulbar conjunctival vessels image.

Bulbar conjunctival blood flow rate is calculated by the blood flow velocity and the vessel diameter, and the formula is

(1) $$\begin{array}{c} Q=V_{s}\frac{\pi D^{2}}{4}. \end{array}$$

In the formula, *Q* is the bulbar conjunctival blood flow rate, *V*_*s*_ is the average blood flow velocity of the cross section of the bulbar conjunctiva vessels, and *D* is the inner diameter of the bulbar conjunctival vessels (the diameter of the vascular cavity). *V*_*s*_ is estimated by the axial blood flow velocity of the bulbar conjunctiva vessels, and the commonly used conversion formula [1] is

(2) $$\begin{array}{c} V_{s}=\left\{\begin{array}{cc} V_{\text{ax}} & ,\;\frac{D}{D_{c}}\leq 0.6,\\ \frac{V_{\text{ax}}}{1.58\left(1-e^{-\sqrt{2D/D_{c}}}\right)} & ,\;\frac{D}{D_{c}}>0.6. \end{array}\right. \end{array}$$

In the formula, *V*_ax_ is the axial blood flow velocity of the bulbar conjunctiva vessels and *D*_*c*_ is the diameter of human erythrocytes, taking 7.65 *μ*m [1]. This conversion formula takes into account the uneven velocity of blood flow across the cross section of the blood vessels.

One way to define bulbar conjunctival vessel density is the ratio of the area occupied by blood vessels in the image to the total area of the image, which can be calculated by counting the number of pixels occupied by blood vessels divided by the total number of pixels. However, this method is affected by vessel diameter. The use of bulbar conjunctival vessel length density, i.e., the length of bulbar conjunctival vessels per unit area [6], can exclude the effect of vessel diameter. Another way is fractal, an algorithm that reflects structural complexity and irregularities, and fractal dimensions can reflect the complexity and density of blood vessels [7]. Liu et al. [8] confirmed that the fractal dimension of the bulbar conjunctival vessels is positively correlated with the bulbar conjunctival vessel density obtained by pixel counting.

In addition to the above four main bulbar conjunctival microcirculation parameters, Cheung et al. [9] summarized 15 identifiable abnormal alterations in bulbar conjunctival microcirculation in diabetic patients, including abnormal vessel diameter, abnormal vascular wall thickness, beading, curvature, congestion, distension, injury, hemosiderin deposition, microaneurysm, abnormal vascular distribution, abnormal arteriovenous ratio, ischemic area, obstruction, intermittent blood flow, and abnormal blood flow velocity, and defined the severity index (SI) of abnormal alterations in the bulbar conjunctival microcirculation, that is, the number of anomalous alterations in the bulbar conjunctival microcirculation above, used for CAIM semiquantitative observation of bulbar conjunctival microcirculation alterations.

The microcirculation parameters of the bulbar conjunctiva are greatly influenced by physiological factors such as respiration and heartbeat, and patients are often allowed to sit still for 10 minutes before measurement [10]. The bulbar conjunctival microcirculation was observed several times a day, and the measured blood flow velocity, vessel diameter [11], and vessel density [12] of the bulbar conjunctiva were stable. In the two observations with a long interval (17 ± 12 weeks apart), vessel density and blood flow rate of the bulbar conjunctiva were still stable [10]. A study on the stability of bulbar conjunctival vessel density in observations with a distant interval is lacking.

The bulbar conjunctival microcirculation is regulated by the nervous and endocrine systems and has a complex self-regulatory mechanism. Alterations in the microcirculation parameters of the bulbar conjunctiva caused by different pathological conditions are often the same, so the alterations in the microcirculation parameters of the bulbar conjunctiva are nonspecific and their significance needs to be discussed under specific pathological conditions. For example, in dry eye, the faster bulbar conjunctival blood flow velocity, the larger bulbar conjunctival vessel diameter, the greater bulbar conjunctival blood flow rate, and the greater bulbar conjunctival vessel density, indicating that the inflammation of the patient's ocular surface is more serious; in diabetes mellitus, a larger SI indicates that the patient has more serious diabetic vasculopathy, and with the progression of diabetic vasculopathy, bulbar conjunctival blood flow velocity, vessel diameter, and vessel density vary differently.

## 3. Bulbar Conjunctival Microcirculation Alterations in Ocular Diseases

### 3.1. Contact Lens Wearing-Related Bulbar Conjunctival Microcirculation Alterations

With the increasing demand for refractive correction, myopia prevention, and control and medical cosmetology, the number of contact lens wearers is increasing. However, adverse effects of contact lenses are issues to be paid close attention to. Conjunctival congestion is one of the most common adverse effects of contact lenses [13]. The existing diagnosis of conjunctival congestion mainly relies on qualitative indicators, which are subjective, such as the degree of congestion and vascular contour clarity. Bulbar conjunctival microcirculation alterations can be used to quantitatively analyze bulbar conjunctival congestion, facilitate its early diagnosis, and correct grading and can be used to further predict adverse effects of contact lens wearing and guide contact lens wearing.

Contact lens wearing causes bulbar conjunctival microcirculation alterations through 2 different mechanisms. One is the direct physical action between the corneal contact lens and the bulbar conjunctiva, such as friction causing bulbar conjunctival hyperplasia and the tear crescent, which mainly acts on the corneal limbus. The limbal SI was significantly higher in patients who wore soft contact lenses (>2 years) than in those who did not wear contact lenses. The results showed that vessel diameter at the limbus was significantly increased, blood flow velocity was significantly decreased, and bulbar conjunctiva microvessel injury, hemosiderin deposition, congestion, intermittent blood flow, and bulbar conjunctiva microvessel curvature were significantly increased [14]. The effect of orthokeratology (Ortho-K) on bulbar conjunctiva microcirculation was similar, and the limbal SI of patients who wore Ortho-K (>1 year) was significantly higher than that of those who did not wear contact lenses [9].

The other is that wearing contact lenses can indirectly cause bulbar conjunctiva microcirculation alterations through compensatory mechanisms for inadequate blood supply to the bulbar conjunctiva in the contact area of the corneal contact lens, such as dilation and reopening of bulbar conjunctival vessels [15]. The bulbar conjunctival blood flow velocity, blood flow rate, vessel diameter, and vessel density in the area without contact with the soft contact lens were significantly higher in the patients wearing contact lens (>6 months) than in controls [16, 17], where blood flow velocity was positively correlated with the length of time per day and the number of days per week that contact lenses were worn [16]. Even after a full night's rest, bulbar conjunctival blood flow velocity, blood flow rate, and vessel density in habitual (>3 years) contact lens wearers were still greater than those in noncontact lens wearers [17], suggesting that contact lens wearing may cause chronic inflammation of the ocular surface and short periods of rest is not enough to restore damage caused by contact lenses. In addition, wearing contact lenses can also cause short-term alterations in the bulbar conjunctival microcirculation parameters. Blood flow velocity, blood flow rate, vessel diameter, and vessel density of bulbar conjunctiva increased after 6 hours of wearing the soft contact lens, regardless of whether the subjects have worn contact lenses previously [2, 15]. Moreover, the comfort degree of contact lens wearers was positively correlated with bulbar conjunctival blood flow velocity and negatively correlated with bulbar conjunctival vessel density [18].

However, there are currently no studies of bulbar conjunctival microcirculation alterations associated with the wearing of rigid gas-permeable contact lenses. In addition, most of the research on the bulbar conjunctival microcirculation alterations associated with the wearing of contact lenses is limited to observation, and there is a lack of exploration of the diagnosis and grading of conjunctival hyperemia using bulbar conjunctival microcirculation alterations.

### 3.2. Dry Eye-Related Bulbar Conjunctival Microcirculation Alterations

Dry eye is a multifactorial ocular surface disease characterized by homeostasis of the tear film and accompanied by symptoms of ocular discomfort, which seriously affects the quality of life. At present, most clinical dry eye examination and diagnostic methods have the limitations of high subjectivity and lack of objective quantitative indicators and analysis. Ocular surface inflammation is one of the main pathophysiological mechanisms of dry eye [19], and its primary clinical manifestation is conjunctival hyperemia. When the ocular surface is inflamed, due to the increase in the secretion of vasomotor substances such as NO, the vessels dilate and congest, bulbar conjunctival vessel diameter and blood flow velocity increase, and if chronic inflammation occurs, vessel density will also increase under the action of angiogenesis factors such as VEGF [20]. The use of bulbar conjunctival microcirculation alterations allows for quantitative analysis of bulbar conjunctival hyperemia, which helps to improve the sensitivity, specificity, and efficiency of dry eye diagnosis [21].

According to Chen et al. [22], blood flow velocity, blood flow rate, vessel diameter, and vessel density of bulbar conjunctiva in patients with dry eye were significantly higher than those in healthy people. Among them, the areas under the curve of the receiver operating characteristic with bulbar conjunctival vessel diameter and blood flow rate as diagnostic indicators of dry eye were 0.861 and 0.856, respectively, comparable with the ocular surface disease index (OSDI) [23] and the noninvasive tear film break-up time [24, 25], indicating that bulbar conjunctival vessel diameter and blood flow rate have good sensitivity and specificity as diagnostic indicators for dry eye. In addition, bulbar conjunctival vessel density in patients with dry eye was positively correlated with their OSDI, which may mean that bulbar conjunctival vessel density can reflect the symptoms and subjective feelings of patients with dry eye [22]. Moreover, patients with dry eye have significantly reduced bulbar conjunctival blood flow velocity, blood flow rate, vessel diameter, and vessel density after receiving local anti-inflammatory therapy [26], which further demonstrated that the bulbar conjunctival microcirculation alterations reflected the severity of ocular surface inflammation and contributed to the monitoring of the effect of dry eye treatment.

### 3.3. Conjunctival Malignant Melanoma- and Conjunctival Nevus-Related Bulbar Conjunctival Microcirculation Alterations

Conjunctival malignant melanoma is a potentially fatal tumor, while conjunctival nevus is a congenital benign hamartoma derived from the neuroectoderm, which is rarely malignant, and the differential diagnosis of the two is difficult, requiring histopathological examination [27] and the difference in the bulbar conjunctival microcirculation alterations at the lesion is one of the potential distinguishing indicators. In the past, fluorescein angiography was used to observe the bulbar conjunctival microcirculation alterations at the lesion, which had the disadvantages of invasive, time-consuming, and qualitative observation.

Brouwer et al. [28] attempted to use OCTA to distinguish conjunctival nevus from conjunctival malignant melanoma. They examined the density and curvature of the bulbar conjunctiva vessels in the lesions of conjunctival nevus, conjunctival malignant melanoma, and primary acquired melanosis and found that there was no significant difference between vessel density at the site of conjunctival malignant melanoma lesion and conjunctival nevus; both of which were lower than the normal vessel density, and the vessels were more curved than the normal bulbar conjunctival vessels, while vessel density at primary acquired melanosis was similar to that at the normal bulbar conjunctiva. Their study failed to distinguish conjunctival nevus from conjunctival malignant melanoma. Future studies using bulbar conjunctival microcirculation alterations to identify conjunctival malignant melanoma and conjunctival nevus could consider exploring more bulbar conjunctival microcirculation parameters or switching to other imaging devices.

### 3.4. Diabetic Retinopathy-Related Bulbar Conjunctival Microcirculation Alterations

Diabetic retinopathy (DR) is the most common retinal vasculopathy and is one of the leading blinding ocular diseases in people over 50 years of age [29]. According to the severity, retinopathy can be divided into nonproliferative diabetic retinopathy (NPDR) and proliferative diabetic retinopathy (PDR). Patients with DR are visually impaired and difficult to reverse, but reasonable interventions can be implemented to stop their progression [30]. Therefore, the prevention and early diagnosis of DR are very important. The gold standard for DR diagnosis is ophthalmic fundus examination, which often requires dilated pupils and is not suitable for large-scale screening [31]. Alterations in the bulbar conjunctival microcirculation reflect the severity of diabetic vasculopathy, with sensitivity and specificity as diagnostic indicators of type 2 diabetes reaching 78.70% and 69.08% [32]. And its observation has the advantages of simple operation, short time consumption, and no need to pretreat patients, and it is promising to be applied to the early diagnosis or large-scale screening of diabetic retinopathy.

Patients with DR have multiple bulbar conjunctival microcirculation alterations. Schuerch et al. [33] found that there was no significant difference between bulbar conjunctival vessel density in no clinically visible diabetic retinopathy (NDR) patients and healthy controls, while DR patients (did not distinguish between NPDR and PDR) had significantly lower bulbar conjunctival vessel density than healthy people. NDR and NPDR patients had larger bulbar conjunctival venule diameter than healthy people [34].

Patterns of alterations in bulbar conjunctival blood flow velocity in DR patients are complex and controversial. Khansari et al. [34] found that the bulbar conjunctival arteriolar blood flow velocity in NDR patients was significantly smaller than that in healthy people, but there was no significant difference between the arteriolar blood flow velocity in NPDR patients and healthy people. In patients with PDR, the bulbar conjunctival arteriolar blood flow velocity was not significantly different from that of healthy people, but the venular blood flow velocity was greater than that of healthy people. Hwang et al. [35] found that the venular blood flow velocity showed a pattern of first increasing and then decreasing in healthy people, diabetic patients without diabetic complications, and diabetic patients with diabetic complications. Both patients with NDR and diabetes without diabetic complications had lower levels of diabetic vasculopathy, but in the two studies described above, the alterations in bulbar conjunctival blood flow velocity in the two studies were reversed, possibly due to the different types of blood vessels observed (arterioles/venules), different blood vessel diameters, or different circumstances of studying ethnicity, age, and whether subjects have other diseases within each group. Despite the controversy, both studies suggested that early diabetic vasculopathy causes alterations in bulbar conjunctival blood flow velocity, which has the potential to screen for early diabetic vasculopathy, particularly retinopathy. Further studies should focus on how to synthesize the bulbar conjunctival microcirculation parameters to improve the sensitivity and specificity of diabetic retinopathy screening. And longitudinal cohort studies are desperately needed to determine whether bulbar conjunctival microcirculation alterations can predict the occurrence of diabetic retinopathy before other abnormalities are found.

## 4. Conclusions

The translucent nature of the bulbar conjunctiva makes it possible to assist in the diagnosis of ocular diseases by assessing bulbar conjunctival microcirculation alterations noninvasively. In recent years, with the continuous emergence and application of new image acquisition devices and image processing techniques, bulbar conjunctival microcirculation has played an important role in the diagnosis of many ocular diseases and has become more and more refined and automated.

There are still some problems with the current study of bulbar conjunctival microcirculation. The vast majority of studies have been limited to the use of bulbar conjunctival microcirculation alterations as a means of basic study, with fewer assessments of their diagnostic potential. There are two main reasons for this; first, a variety of diseases and physiological states may trigger bulbar conjunctival microcirculation alterations in a similar way, which makes the bulbar conjunctival microcirculation alterations cannot be independently used as a diagnostic indicator of a disease, but only as an auxiliary diagnostic indicator or grading indicator. In addition, the data obtained by different imaging equipment, image processing methods, and algorithms are not uniform, and there is no standardized procedure for bulbar conjunctival microcirculation exploration, which makes the data obtained by different laboratories not comparable.

There is still a wide range of exploration space for research on bulbar conjunctival microcirculation alterations. It will be a series of emerging fields to study and analyze the differences between multiple imaging equipment, image processing methods, and algorithms, update imaging equipment and algorithms, and concrete bulbar conjunctival microcirculation alterations as indicators for ocular diseases with large-scale research.
